This article has been retracted.

# Diagnostic Value of Echocardiography Combined with Serum h-FABP and cTnI in Myocardial Infarction and Its Evaluation Value in Left Ventricular Function

**DOI:** 10.1155/2022/8809708

**Published:** 2022-05-24

**Authors:** Yanling Miao, Ying Liu, Chao Liu, Lei Yao, Xiaoning Kang, Maoting Lv

**Affiliations:** Department of Ultrasound II, Cangzhou Central Hospital, Cangzhou, China

## Abstract

**Objective:**

To explore the value of color Doppler echocardiography (CDE) combined with serum heart-type fatty acid-binding protein (h-FABP) and cardiac troponin I (cTnI) in the diagnosis of myocardial infarction and its evaluation value in left ventricular function.

**Methods:**

A total of 44 patients with myocardial infarction who were treated in Cangzhou Central Hospital from October 2018 to February 2020 were included in the observation group, and 45 healthy subjects were included in the control group. The serum h-FABP and cTnI levels of the two groups were compared and analyzed. The coincidence rate of echocardiography plus serum h-FABP and cTnI for single diagnosis and combined diagnosis was analyzed. The left ventricular function indexes of patients with myocardial infarction in different cardiac function grades were compared, including left ventricular end-diastolic diameter (LVEDD), left ventricular end-systolic diameter (LVESD), left ventricular end-systolic volume (LVESV), left ventricular end-diastolic volume (LVEDV), stroke volume (SV), cardiac index (CI), and the ratio of peak velocity blood flow from left ventricular relaxation in early diastole to peak velocity flow in late diastole (E/A). The value of echocardiography combined with serum h-FABP and cTnI in the left ventricular function in patients with myocardial infarction was analyzed.

**Results:**

The levels of serum h-FABP and cTnI in the observation group were significantly higher than those in the control group (*P* < 0.05). CDE plus serum h-FABP and cTnI was associated with significantly higher sensitivity, specificity, and accuracy in diagnosing myocardial infarction versus single detection (*P* < 0.05). The LVEDV, SV, and CI parameters were similar in patients with different cardiac function grades (*P* > 0.05). Compared with cardiac function grades I and II, the level of LVEF in patients with myocardial infarction in grades III and IV of cardiac function decreased, while the levels of LVEDD, LVESD, LVESV, and E/A increased (*P* < 0.05). The levels of serum h-FABP and cTnI in patients with myocardial infarction increased with the increase of cardiac function grades (*P* < 0.05).

**Conclusion:**

Patients with myocardial infarction show high levels of h-FABP and cTnI, and CDE plus the detection of serum h-FABP and cTnI levels can significantly improve the detection accuracy and effectively evaluate the left ventricular function of patients with myocardial infarction, with a certain predictive value for cardiac function grading in myocardial infarction.

## 1. Introduction

Acute myocardial infarction (AMI) is myocardial necrosis caused by acute and persistent ischemia and hypoxia of the coronary artery, with clinical manifestations of arrhythmia, acute circulatory dysfunction, chest pain, heart failure, and even shock, which impose a substantial threat on the life of patients [1, 2]. Patients with AMI are usually accompanied by heart failure in which ventricular filling or ejection is impaired due to structural or functional abnormalities of the heart. Accurate assessment of cardiac function is of great significance for the treatment and prognosis of patients with myocardial infarction [3, 4]. There are currently many clinical methods for assessing cardiac function, including echocardiography, serological markers, and cardiac function classification by the New York Heart Association (NYHA), among which the NYHA cardiac function classification is widely used in clinical practice yet lacks quantitative indicators [5, 6]. Color Doppler echocardiography (CDE) is an important auxiliary method for evaluating cardiac structure and function. Despite its easy operation and higher safety profiles, image acquisition is easily affected by factors such as heart rate [7]. Heart-type fatty acid-binding protein (h-FABP) is abundant in the myocardial cytoplasm, and the degree of elevation can reflect the severity of myocardial damage [8, 9]. It is a new type of intracellular fatty acid carrier protein with high sensitivity for the diagnosis of myocardial damage. Cardiac troponin (cTnI) has high specificity for the detection of cardiac function and is the primary marker for cardiac damage [10, 11]. The innovation of this study is the use of echocardiography. Early diagnosis of myocardial infarction using ECG has a high rate of missed diagnosis and misdiagnosis, and it usually requires the combination of clinical manifestations for AMI diagnosis, which delays the treatment. In the present study, 44 patients with myocardial infarction in Cangzhou Central Hospital were recruited to explore the value of CDE plus serum h-FABP and cTnI in the diagnosis of myocardial infarction and the evaluation of left ventricular function.

## 2. Study Population and Methods

### 2.1. Participants

Between October 2018 and February 2020, a total of 44 patients with myocardial infarction who were treated in the Cangzhou Central Hospital were included in the observation group, and 45 healthy subjects were included in the control group. The baseline data of the observation group (23 males and 21 females, aged 33–75 years, with an average age of (54.57 ± 10.38) years, 20 cases of inferior wall and 24 cases of anterior wall in terms of infarction site, 11 cases of grade I, 12 cases of grade II cases, 12 cases of grade III, and 9 cases of grade IV in terms of cardiac function classification) were comparable with those of the control group (25 males and 20 females, aged 33–75 years, with an average age of (54.61 ± 10.29) years) (*P* > 0.05, Tables 1 and 2). All patients voluntarily participated in the present study and signed informed consent prior to the enrollment, and this study was reviewed and approved by the Ethics Committee of the Cangzhou Central Hospital. The ethics approval number is 2017-12-11.

### 2.2. Inclusion and Exclusion Criteria

Inclusion criteria were as follows: the patients in the observation group met the diagnostic criteria of Guidelines for the Diagnosis and Treatment of Acute Myocardial Infarction: ① clinical manifestations of myocardial ischemia, ② pathological Q wave on ECG, and ③ confirmed by coronary angiography. Any one of the above conditions with an increase in serum myocardial enzymes more than 2 times normal can be diagnosed as myocardial infarction. Exclusion criteria were as follows: patients with recent cerebral embolism, pulmonary embolism, and lower extremity venous embolism; with renal insufficiency; and with malignant tumors and abnormal consciousness.

## 3. Methods

The detection method of CDE plus serum h-FABP and cTnI: 3 ml of venous blood was collected from the patients in the observation group when chest pain occurred, and 3 ml of fasting venous blood was collected from the patients in the control group. The venous blood samples were centrifuged to obtain the supernatant, placed in a dry and clean test tube, and stored in a −20°C refrigerator for inspection. Serum h-FABP level was determined by the enzyme-linked immunosorbent sandwich method using a Beckman AU5800 automatic biochemical analyzer. Serum cTnl level was determined by a Beckman ACCESS 800 automatic chemiluminescence immunoassay analyzer. Positive criteria: h-FABP level >2.50 ng/ml; cTnl level >0.35 ng/ml. The frequency of the CDE probe is 2–4 MHz, and the positive criteria are as follows: the segmental ventricular wall in the infarcted area is thinned and the ventricular wall motion is contradictory, weakened, or disappeared, and the myocardial echo was weakened or increased. Positive is considered if the case of any positive results of one of the above examinations.

Detection of parameters related to left ventricular function by CDE: the cardiac function grades of all subjects were assessed by two attending physicians in cardiology with consistent determination. Using GEViVidE9 and PhilipsIE33 cardiac color Doppler ultrasound diagnostic equipment, M5ScD, and S5-1 transthoracic probe, subjects were placed in the supine, semirecumbent, or lateral position, and LVEF, left ventricular end-diastolic diameter (LVEDD), left ventricular end-systolic diameter (LVESD), left ventricular end-systolic volume (LVESV), left ventricular end-diastolic volume (LVEDV), stroke volume (SV), cardiac index (CI), and the ratio of peak velocity blood flow from left ventricular relaxation in early diastole to peak velocity flow in late diastole (E/A) were measured as per the guidelines of the American Society of Echocardiography.

### 3.1. Treatment Methods

Patients in both groups were given percutaneous coronary intervention (PCI) and medication treatment. After the patients were diagnosed with AMI, they were given oral aspirin enteric tablets at an initial dose of 300 mg/d, maintained at a dose of 10 mg/d for the lifetime, and received PCI for treatment.

### 3.2. Statistical Analysis

All data analyses were performed with SPSS 20.0 software. Measurement data were expressed as (*x* ± *s*), one-way analysis of variance was used for comparison amongst multiple groups, and the independent samples *t* test was used for comparison between two groups. Enumeration data were expressed as number of cases (rate), and the chi-square test was used for the comparison. Differences were considered statistically significant at *P* < 0.05.

## 4. Results

### 4.1. Comparison of Serum h-FABP and cTnI Levels

The levels of serum h-FABP and cTnI in the observation group were significantly higher than those in the control group (*P* < 0.05).

### 4.2. Diagnostic Results of Echocardiography Combined with Serum h-FABP and cTnI Levels

The sensitivity, specificity, and accuracy of ECD combined with serum h-FABP and cTnI levels in diagnosing patients with myocardial infarction were significantly higher than those of single detection and diagnosis (*P* < 0.05), as given in Tables 3 and 4.

### 4.3. Comparison of Echocardiographic Parameters in Patients with Myocardial Infarction with Different Cardiac Function Grades

The LVEDV, SV, and CI parameters were similar in patients with different cardiac function grades (*P* > 0.05). Compared with cardiac function grades I and II, the level of LVEF in patients with myocardial infarction in grades III and IV of cardiac function decreased, while the levels of LVEDD, LVESD, LVESV, and E/A increased (*P* < 0.05).

### 4.4. Comparison of Serum h-FABP and cTnI Levels in Patients with Myocardial Infarction with Different Cardiac Function Grades

The levels of serum h-FABP and cTnI in patients with myocardial infarction increased sequentially with the increase of cardiac function grades (*P* < 0.05), as given in Table 5.

## 5. Discussion

Myocardial infarction features rapid progression and high clinical mortality, with characteristics of the thinning of the systolic ventricular wall. Its main influencing factors comprise unstable emotions, overeating, constipation, and cold stimulation, seriously threatening the health of patients [12, 13]. Hence, efficient diagnostic methods are essential to timely prevent and treat myocardial infarction. Patients with myocardial infarction are usually diagnosed by clinical manifestations and ECG changes, but the rate of missed diagnosis and misdiagnosis is high. The myocardial injury markers serum cTnI and serum h-FABP are common indicators for clinical diagnosis of myocardial infarction. h-FABP is a soluble cytoplasmic protein mainly distributed in cardiomyocytes. It is highly sensitive in the early stage of myocardial infarction and can rapidly increase within 1-2 hours of onset. ECD is an important auxiliary method for evaluating cardiac structure and function with the simple clinical operation and high in safety and thus serves as an efficient diagnostic method. Myocardial infarction is mainly characterized by thinning and strengthening of myocardial echo.

The results of the present study showed that the serum h-FABP and cTnI levels in patients with myocardial infarction were significantly higher than those in healthy subjects; the sensitivity, specificity, and accuracy of CDE combined with serum h-FABP and cTnI levels in diagnosing patients with myocardial infarction were significantly higher than those of every single detection and diagnosis. The results indicate that serum h-FABP and cTnI levels are efficient indicators for the clinical diagnosis of myocardial infarction, and the diagnostic results of CDE plus serum h-FABP and cTnI levels are more accurate. CDE can evaluate a patient's cardiac function and the desynchrony of myocardial phase motion. Among cardiac function-related parameters, LVEF, LVESD, and LVESV can reflect left ventricular systolic function in patients with myocardial infarction, and LVEDD, LVEDV, and E/A can evaluate the left ventricular diastolic function [14, 15]. Ding et al. have found that CDE can better evaluate left ventricular morphology and diastolic function in patients with left ventricular diastolic myocardial infarction, and compared with healthy people, patients with left ventricular diastolic myocardial infarction have significantly higher left ventricular posterior wall thickness, LVEDD, and E/A [16]. Gong et al. reported that compared with healthy subjects, patients with myocardial infarction have significantly higher LVESD and LVESV [17, 18].

Here, the levels of LVEDD, LVESD, LVESV, and E/A increased with the deterioration of cardiac function and were significantly correlated with the cardiac function classification of patients with myocardial infarction, suggesting a relation of the gradual expanded left ventricle of patients with myocardial infarction to compensatory blood supply [19] and also to the relative mitral valve insufficiency in patients with cardiac function class III and IV. LVEF, LVEDD, LVESD, LVESV, and E/A show great potential as objective indicators for predicting cardiac function class [20, 21]. However, the Doppler frequency is affected by the coordination of the ventricle, and the analysis of the local myocardial activity disorder requires more understanding of the specific clinical situation.

h-FABP is a heart-specific fatty acid-binding protein that is widely present in cardiomyocytes with a high diagnostic value for myocardial damage. Cai et al. reported that serum h-FABP and hs-cTnI levels increased with the severity of asphyxia in children, and their levels in children with severe asphyxia complicated with myocardial damage were significantly higher than those in children without myocardial damage. The expression levels of the two have a certain diagnostic value for neonatal asphyxia complicated with myocardial damage. cTnI is a myocardial-specific structural protein, 97% of which exists in the cytoplasm of myocardial cells in the form of complexes. It participates in myocardial contractility with myocardial calcium ions. When myocardial cells are damaged or necrotic, cTnI will be released in blood, with the increase of its level proportional to the severity of myocardial damage and is considered an important reference index for clinical detection of myocardial damage, with high tissue specificity and sensitivity. The present study found that there was no significant difference in LVEDV, SV, and CI parameters in patients with different cardiac function grades; compared with cardiac function grades I and II, the level of LVEF in patients with myocardial infarction in grades III and IV of cardiac function decreased, while the levels of LVEDD, LVESD, LVESV, and E/A increased; the levels of serum h-FABP and cTnI in patients with myocardial infarction increased sequentially with the increase of cardiac function grades, suggesting the value of LVEF, LVEDD, LVESD, LVESV, E/A, serum h-FABP, and cTnI levels in evaluating the cardiac function classification of patients with myocardial infarction. The limitation of this study is the absence of a diagnostic effect test for these indicators to clarify their diagnostic efficacy. In the future, a detailed diagnostic efficacy test will be performed to allow for early diagnosis of AMI.

Traditional Chinese medicine treatment of AMI can protect damaged myocardium and improve myocardial function through local relief and systemic regulation. The patients were classified into Qi deficiency and blood stasis type, Qi deficiency and phlegm stasis type, heart Qi deficiency type, and heart Yang deficiency type as per the “Criteria Related to the Diagnostic Efficacy of Chinese Medicine Evidence” [1] and the relevant experience of AMI diagnosis. According to the general principle of “unblocking as the main treatment and tonification as supplement before surgery, and tonification as the main treatment and unblocking as supplement after surgery,” for patients with Qi deficiency and blood stasis type, 20 mL/d of Astragalus injection (equivalent to 40 g of the raw drug Astragalus) and compound Danshen injection (2 mL/stem, equivalent to raw drug containing 2 g each of Danshen and Radix et Rhizoma) were given intravenously to invigorate blood, benefit Qi, and clear stasis; for patients with Qi deficiency and phlegm stasis type, Astragalus injection 20 mL/d (equivalent to 40 g of raw Astragalus) was given intravenously to invigorate blood, benefit Qi, resolve phlegm, and clear the blood circulation; intravenous injection of Astragalus injection 20 mL/d (equivalent to 40 g of raw Astragalus) for patients with deficiency of heart Qi; ginseng and *Sophora* injection (red ginseng and black *Sophora* extracts, with main ingredients of ginsenoside >0.5 mg/mL and aconitine) was given intravenously for patients with the heart Yang deficiency type.

## 6. Conclusion

Patients with myocardial infarction show high levels of h-FABP and cTnI, and CDE plus the detection of serum h-FABP and cTnI levels can significantly improve the detection accuracy and effectively evaluate the left ventricular function of patients with myocardial infarction, with a certain predictive value for cardiac function grading in myocardial infarction.

## Figures and Tables

**Table 1:** Comparison of baseline features of the two groups of patients (*n* (%)).

	Observation group (*n* = 44)	Control group (*n* = 45)	*t*/*x*^2^	*P*
Gender			0.096	0.756
Male	23	25		
Female	21	20		
Mean age	54.57 ± 10.38	54.61 ± 10.29	−0.018	0.986
Infarct site			—	—
Lower wall	20	—		
Front wall	24	—		
Cardiac function grades			—	—
I	11			
II	12			
III	12			
IV	9			

**Table 2:** Comparison of serum h-FABP and cTnI levels between the two groups (*x* ± *s*).

Groups	*n*	h-FABP (ng/ml)	cTnI (ng/ml)
Observation group	44	79.21 ± 9.35	31.28 ± 9.84
Control group	45	1.72 ± 0.51	0.18 ± 0.06
*t*	—	55.518	21.204
*P*	—	<0.001	<0.001

**Table 3:** Echocardiography, serum h-FABP, and cTnI levels alone and hybrid detection of myocardial infarction (*n* (%)).

Indexes	Sensitivity	Specificity	Accuracy
h-FABP	77% (34/44)	73% (33/45)	75% (67/89)
cTnI	75% (33/44)	76% (34/45)	75% (67/89)
ECD	80% (35/44)	71% (32/45)	75% (67/89)
Hybrid detection	95% (42/44)	93% (42/45)	94% (84/89)
*x* ^2^/*P*, h-FABP-hybrid detection	6.175/0.013	6.48/0.011	12.618/<0.001
*x* ^2^/*P*, cTnI-hybrid detection	7.311/0.007	5.414/0.02	12.618/<0.001
*x* ^2^/*P*, hybrid detection	5.091/0.024	7.601/0.006	12.618/<0.001

**Table 4:** Comparison of echocardiographic parameters in patients with myocardial infarction with different cardiac function grades (*x* ± *s*).

Cardiac function grades	*n*	LVEF (%)	LVEDD (mm)
I	11	49.15 ± 9.13	49.81 ± 6.32
II	12	48.28 ± 8.05	49.74 ± 6.28
III	12	42.36 ± 7.25^①②^	60.06 ± 11.33^①②^
IV	9	37.62 ± 5.66^①②③^	61.48 ± 11.56^①②^
*F*	—	4.976	5.284
*P*	—	0.005	0.004
Cardiac function grades	*n*	LVESD (mm)	LVESV (mL)
I	11	33.76 ± 6.95	1.52 ± 0.27
II	12	33.79 ± 7.01	1.64 ± 0.28
III	12	48.24 ± 11.30^①②^	1.84 ± 0.36^①②^
IV	9	50.53 ± 11.42^①②^	1.92 ± 0.26^①②^
*F*	—	10.162	3.933
*P*	—	<0.001	0.015
Cardiac function grades	*n*	LVEDV (mL)	SV (mL)
I	11	91.64 ± 33.56	49.12 ± 19.30
II	12	98.69 ± 33.21	51.84 ± 21.28
III	12	120.17 ± 58.55	58.97 ± 28.03
IV	9	117.43 ± 43.38	53.29 ± 17.66
*F*	—	1.134	0.405
*P*	—	0.347	0.75
Cardiac function grades	*n*	CI	E/A
I	11	2.16 ± 0.86	1.18 ± 0.23
II	12	2.21 ± 0.91	1.21 ± 0.27
III	12	2.69 ± 0.82	1.96 ± 0.32^①②^
IV	9	2.56 ± 0.66	2.04 ± 0.34^①②^
*F*	—	1.123	27.752
*P*	—	0.351	<0.001

^①^Compared with grade I, *P* < 0.05. ^②^Compared with grade II, *P* < 0.05. ^③^Compared with grade III, *P* < 0.05.

**Table 5:** Comparison of serum h-FABP and cTnI levels in patients with myocardial infarction with different cardiac function grades (*x* ± *s*).

Cardiac function grades	*n*	h-FABP (ng/ml)	cTnI (ng/ml)
I	11	4.64 ± 1.16	0.92 ± 0.18
II	12	4.94 ± 1.22^①^	3.15 ± 0.61^①^
III	12	9.38 ± 1.82^①②^	8.63 ± 1.74^①②^
IV	9	9.83 ± 1.96^①②^	12.78 ± 2.54^①②③^
*F*	—	34.638	131.032
*P*	—	<0.001	<0.001

^①^Compared with grade I, *P* < 0.05. ^②^Compared with grade II, *P* < 0.05. ^③^Compared with grade III, *P* < 0.05.

## Data Availability

The data generated or analyzed during this study are included within the article.
